# Investigation on the Operation Status of Community-Based Rehabilitation Station in a District of Chongqing

**DOI:** 10.1155/2021/6044923

**Published:** 2021-11-23

**Authors:** Jingxuan Shang

**Affiliations:** Chongqing City Management College, Chongqing 401331, China

## Abstract

**Objective:**

Investigate and analyze the current operation status of the community-based rehabilitation station in a district of Chongqing to provide some reference schemes for improving the construction of the community-based rehabilitation system for Chongqing.

**Methods:**

Self-designed questionnaires were issued to 36 community-based rehabilitation stations in a district of Chongqing to investigate the human resources status, service projects, service methods, and other aspects of the community-based rehabilitation stations.

**Results:**

The community-based rehabilitation station lacks the participation of medical rehabilitation personnel, and only 33.3% of the community-based rehabilitation stations are composed of multidisciplinary human resources of medical and community staff. Community-based rehabilitation services focus on supply education and publicity (86.11%), and rehabilitation treatment services are not fully involved in the community-based rehabilitation service (44.44%). The methods of community-based rehabilitation services are mainly posters and other publicity activities (94.44%), and the community-based rehabilitation service methods are not highly goal-oriented.

**Conclusion:**

The survey found some problems to be improved in the construction and operation of grass-roots community-based rehabilitation stations in Chongqing. Community-based rehabilitation stations should enrich the human resources and technology of medical rehabilitation, become an extension of the restoration of community health institutions, and promote the high-quality development of community-based rehabilitation.

## 1. Introduction

As an important platform for the rehabilitating of the disabled in China, the community-based rehabilitation station is the extension of the restoration of medical and health institutions outside the hospital. It plays an essential role in community-based rehabilitation with its nearby and local advantages. Since 2004, Chongqing Disabled Persons' Federation has built thousands of community-based rehabilitation stations and introduced relevant measures and policies to ensure the operation of community-based rehabilitation stations. However, in the further work of the Chongqing Disabled Persons' Federation, there is still a lack of the actual process of the data of the community-based rehabilitation station. The purpose of this study is to investigate the progress of community-based rehabilitation stations for the disabled in a district of Chongqing, discuss the construction and service of community-based rehabilitation stations, and provide a basis for the improvement and improvement of community-based rehabilitation services in Chongqing.

## 2. Objects and Methods

### 2.1. Object of Study

In December 2020, the institutional establishment, operation, and business development of 36 community-based rehabilitation stations in Chongqing were investigated.

### 2.2. Research Methods

A self-designed community-based rehabilitation station operation questionnaire and face-to-face survey method were adopted. Fill in and report by the person in charge of each community-based rehabilitation station in a district of Chongqing.

### 2.3. Quality Control

First, the questionnaire and the instructions for filling the form were carefully formulated. Second, concentrate on training the investigators and explain the questionnaire in detail to reach the consensus on the key issues that need to be paid attention to in the survey. Investigators shall be appointed after passing the simulation survey and test. Third, carry out investigation, on-site guidance, spot check, and verify data.

36 questionnaires were sent out, and 36 were effectively received with an effective recovery rate of 100%. All the questionnaires fill in independently and recover on the spot after the questionnaire is completed.

### 2.4. Statistical Method

Excel software was used to input and handle the data, and two investigators were in charge of inputting and proofreading data. Frequency and percentage were mainly used to describe the data.

## 3. Results

### 3.1. The Running Time of Community-Based Rehabilitation Stations

There are 11 (30.56%) community-based rehabilitation stations that have been operating for over ten years, 1 (2.78%) community-based rehabilitation station that has been working for five years (inclusive) to 9 years, 1 (2.78%) community-based rehabilitation station that has been working for four years, 5 (13.89%) community-based rehabilitation stations that have been working for three years, 15 (41.67%) community-based rehabilitation stations that have been working for two years, and 3 (8.33%) other that have been working for one year. Overall, a large proportion of the community-based rehabilitation stations in a district of Chongqing have been working for three years or less (63.89%), and their operating time is relatively short (Table 1).

### 3.2. Human Resources of Community-Based Rehabilitation Station

Among the human resources composition structures of the community-based rehabilitation stations, 5 (13.89%) were composed solely of medical staff. 12 (33.33%) community-based rehabilitation stations were composed of medical and community staff, and 19 (52.78%) others were composed solely of community staff. Professional medical and health human resources are less involved in community-based rehabilitation stations (Table 2).

### 3.3. Service Items of Community-Based Rehabilitation Station

Among the service items of community-based rehabilitation stations, education and publicity services (86.11%) were the most, followed by auxiliary equipment fitting (69.44%), rehabilitation treatment (44.44%), referral (38.89%), public social affairs (25.00%), and vocational rehabilitation services not carried out. Rehabilitation treatment and referral services accounted for relatively few. High-level and targeted rehabilitation services in community-based rehabilitation stations are rather inadequate (Table 3).

### 3.4. Service Mode of Community-Based Rehabilitation Station

Among the service modes of community-based rehabilitation stations, the focus was on posters (94.44%) and collective activities (61.11%), followed by in-station face-to-face service (50.00%) and door-to-door service (41.67%), while online interactive rehabilitation services were not carried out (Table 4).

### 3.5. Factors That Restrict the Operation of Community-Based Rehabilitation Stations

Among the factors restricting the operation of community-based rehabilitation stations, small site area (41.67%) is considered the main factor limiting the procedure, in turn, understaffed (25.00%), others (22.22%), insufficient funding (19.44%), poor awareness of disabled rehabilitation (13.89%), lack of equipment (11.11%), lack of relevant knowledge or skills (8.33%), and lack of assessment mechanism (5.56%) (Table 5).

## 4. Discussion

Rehabilitation is the most immediate, urgent, and realistic need of the disabled, patients with chronic diseases, and the elderly. It plays a vital role in dealing with the aging of the population and ensuring the health of the whole people. To achieve the sustainable development goal in 2030, rehabilitation services need to be strengthened to expand rehabilitation as a health strategy related to all humankinds in the whole life cycle and national health cover and meet the growing demand for rehabilitation [1].

Rehabilitation services run throughout the process of healthcare services, and efforts should be made to improve its quality, accessibility, and affordability [2]. Community-based rehabilitation has the advantages of easy convenience, low price, and easy acceptance. Promoting low-cost and extensive community-based rehabilitation is a crucial way to achieve fair and accessible rehabilitation services [3].

To meet to address the growing demand for rehabilitation, the plan for a Healthy China 2030 proposes that it is necessary to improve the medical and health service system and promote the extension of medical and health services to communities and families. The World Health Organization (WHO) also pointed out that rehabilitation should be included in the health service system, and hospitals and districts should provide rehabilitation services and reasonably allocate health service resources [4].

Feng bo Liu proposed that different categories of disabled people are different in the rehabilitation needs, and the particularity of the needs of the different types disabled should be considered when providing rehabilitation services [5]. The rehabilitation needs of the disabled in China mainly include medical services and assistance, assistive devices, rehabilitation training and services, help for the poor disabled people, barrier-free facilities, information accessibility, and other rehabilitation needs [1]. To meet the differentiated health needs of different groups of people at different life stages, we should strive to promote the deep integration of rehabilitation and medical treatment and form a solid synergy to maintain and promote health [3].

Community-based rehabilitation station is the central position and window of the disabled community-based rehabilitation and window. According to this survey, the community-based rehabilitation station has certain hardware facilities (such as site and rehabilitation equipment) and has achieved inevitable development, but there are some problems.

According to this survey, the construction of the community-based rehabilitation station has been equipped with particular hardware facilities (such as site and rehabilitation equipment) and achieved certain development, but there are some problems. First, the structure of human rehabilitation resources is unreasonable. The operation of the community-based rehabilitation station mainly depends on the community staff, and the intervention of medical rehabilitation services is insufficient. Second, the supply of rehabilitation services focuses on posting posters and other areas of education or publicity activities. Finally, without the support of rehabilitation professionals and technical personnel, rehabilitation services are not strongly targeted. It is challenging to ensure high-quality community-based rehabilitation services, the stability of the work, and the sustainability of the service. Nonprofessional rehabilitation services cannot effectively solve the rehabilitation problem of the disabled.

In the document on accelerating the development of the work of rehabilitation medicine, it is proposed to actively develop community-based and home-based rehabilitation medical care and support grass-roots medical institutions to enrich and innovate rehabilitation medical service models. Community-based rehabilitation stations, which are an essential carrier of rehabilitation into communities and services to families, should be integrated with grass-roots health institutions and become the “rehabilitation outpatient service” of grass-roots health institutions or the extension of medical services. Although the technical level of healthcare workers in grass-roots community health service centers (station) and rural towns generally remains to be improved, grass-roots medical staff have apparent advantages in ensuring residents' elderly care and rehabilitation. Through technical training and service model innovation, they can become the backbone of the combination of medical care and long-term care services, which is not only possible but also necessary [6].

The development goal of community health service in China is the family doctor system [7]. The elderly, the patients with chronic diseases, the disabled, and other vulnerable groups are inconvenient to walk, and it is difficult to go out for medical treatment. The use of family doctor contract service is conducive to solve the complex problems of vulnerable groups such as medical access. Community-based rehabilitation stations also need to further enrich the medical professional and technical resources. It can give full play to the role of “Internet+,” home beds, and door-to-door visits to the community and home and provide home rehabilitation medical care, day rehabilitation training, rehabilitation guidance, and other services for the elderly, patients with chronic diseases, people with severe disabilities, and other people in urgent need of rehabilitation services.

To comprehensively promote the construction of healthy China and actively respond to the aging population and other national strategies, the construction of community-based rehabilitation urgently needs health management department to include community-based rehabilitation medical facilities and talents such as community-based rehabilitation stations into the construction planning of the medical and health service system, improve the functions of primary health service institutions integrating prevention, medical treatment, rehabilitation and healthcare, integrate existing resources, and enhance the rehabilitation capacity of community health institutions based on community-based rehabilitation stations.

## 5. Conclusion

Community-based rehabilitation stations are the main position and link for the elderly, chronic disease patients, the disabled, and other vulnerable groups to obtain community-based rehabilitation services. At present, the human resources and technology of medical rehabilitation of community-based rehabilitation stations should be enriched, so that the community-based rehabilitation stations can become the carrier of grass-roots health institutions to the community and families and open up the last “kilometer” of community-based rehabilitation, so as to achieve the accessible and high-quality development of community-based rehabilitation services.

## Figures and Tables

**Table 1:** The running time of the community-based rehabilitation station (*n* = 36).

The running time	Number	Proportion (%)
≥10 years	11	30.56
5–9 years	1	2.78
4 years	1	2.78
3 years	5	13.89
2 years	15	41.67
1 year	3	8.33

**Table 2:** Human resource structure of community-based rehabilitation stations (*n* = 36).

Human resource structure	Number	Proportion (%)
Pure professional medical personnel	5	13.89
A mix of medical and community staff members	12	33.33
Simple community worker	19	52.78

**Table 3:** Service items of the community-based rehabilitation station (*n* = 36).

Service project	Number	Proportion (%)
Rehabilitation treatment	16	44.44
Education and publicity	31	86.11
Vocational rehabilitation	0	0
Social and public affairs	9	25
Assistive devices fit	25	69.44
Referral	14	38.89

**Table 4:** Service modes of community-based rehabilitation stations (*n* = 36).

Service mode	Number	Proportion (%)
Door-to-door service	15	41.67
Posters and other publicity	34	94.44
Collective activity	22	61.11
Face-to-face service in the station	18	50
Online interactive rehabilitation services	0	0

**Table 5:** Factors restricting the operation of community-based rehabilitation stations (*n* = 36).

Factors	Quantity	Scale (%)
Lack of relevant knowledge or skills	3	8.33
Lack of equipment	4	11.11
Small site area	15	41.67
Insufficient funded	7	19.44
The short of hands	9	25
Lack of the assessment mechanism	2	5.56
Poor awareness of disabled	5	13.89
Others	8	22.22

## Data Availability

The data used to support the findings of this study are available from the corresponding author upon request.
